This article has been retracted.

# An osteotomy anterolateral approach for lateral tibial plateau fractures merged with relatively simple and intact posterolateral corner displacement

**DOI:** 10.1186/1749-799X-9-26

**Published:** 2014-04-15

**Authors:** De-peng Meng, Tian-wen Ye, Ai-min Chen

**Affiliations:** 1 Department of Orthopedic Surgery, Changzheng Hospital, The Second Military Medical University, 415 Fengyang Road, Huangpu District, Shanghai 200003, China

**Keywords:** Lateral tibial plateau fractures, Posterolateral corner displacement, Anterolateral approach, Indication and techniques

## Abstract

**Introduction:**

This study investigates the safety and efficacy of anterolateral (AL) osteotomy for the treatment of lateral tibial plateau fractures merged with relatively simple and intact posterolateral (PL) corner displacement and screens applicable patients.

**Methods:**

Totally, 11 patients with lateral tibial plateau fractures involving the PL corner were included in this study. Of them, seven patients sustained their injuries from motor vehicle accidents (MVAs), three from sports and one from fall from height. All of them received open reduction and internal fixation through the AL approach. Operation time, incision length, range of motion (ROM), Hospital for Special Surgery (HSS) knee score, time of union and complications were retrospectively reviewed. Tibial plateau angle (TPA), lateral posterior slope angle (PSA) and articular step-off reduction after surgery were examined by a radiograph technique.

**Results:**

Statistically, the means of operation time, incision length, ROM and follow-up period were 82 min, 11 cm, 97° and 27 months, respectively. Three patients had slight complications: superficial infection, hardware irritation and secondary valgus deformity, without severe neural or vascular injuries, which revealed the safety and efficacy of the PL treatment. The average HSS knee score was 91.2 (range 86–96). Reduction (mean TPA 87.2° and mean PSA 8.3°) was satisfactory in 10 patients, except for one patient with a radiographic articular step-off of 5 mm (case 10).

**Conclusions:**

The AL approach is safe and effective for lateral tibial plateau fractures involving the PL corner, especially for fractures merged with simple and intact PL corner displacement (depression and/or split).

## Introduction

A posterolateral (PL) tibial plateau fracture is an unusual type of fracture which is rarely reported in the past [1]. Based on the classification system of the AO Foundation and Orthopaedic Trauma Association (AO/OTA) [2], a PL tibial plateau fracture can be classified into 41-B1.1(4), 41-B3.1(2) and 41-B2.2(4). This fracture has the following features: the mainly displaced fragment is located at the posterior half of the lateral condyle and/or a fracture line impacts the posterior aspect of the lateral plateau [3].

According to the classification, the suggested treatment of PL plateau fractures is the use of the posterior approach for anatomical reduction and rigid fixation, as the posterior approach is believed to be easy for full exposure and surgical manipulations [4-8]. The posterior approach can provide direct exposure of the fracture, enabling fracture reduction under visualisation and buttress plate fixation. However, many important nerves and vessels distribute just in the surgical area, such as the common peroneal nerve at the posterior aspect of the biceps femoris muscle, the popliteal vessels, the saphenous nerve at the posterior aspect of the medial plateau, the medial sural cutaneous nerve and the tibial nerve in the popliteal fossa [6]. Therefore, the posterior approach can lead to considerable risks of soft tissue injuries, such as paresthesia (12.5%–60%) [5,9,10], skin complications (14%) [11], vascular injury (20%) [9,12] and flexion contracture (50%) [10,13].

Based on anatomical features, the anterior approach is much safer than the posterior approach, because there is no important neurovascular structure in the surgical area. In recent years, the anterior approach has been successfully used to treat PL tibial plateau fractures and also obtained good clinical outcomes [3]. However, the related indications and technical essentials are still unclear. Actually, we agree that the anterolateral (AL) approach may be a safe and effective therapy for the treatment of PL tibial plateau fractures in a certain group of patients as the literature reported. In this study, we want to conclude our patient inclusion criteria and the technical essentials of the AL approach for the treatment of PL tibial plateau fractures and further to investigate the safety and effectiveness of the isolated AL approach for such fractures.

## Methods

### The inclusion criteria and screening of proper patients

The inclusion criteria of the fractures for this study were as follows: (i) a fresh lateral tibial plateau fracture classified as 41-B1.1(4), 41-B2.2(3), 41-B2.2(4), 41-B3 or 41-B3.1(2) according to the AO/OTA classification system (within 21 days); (ii) a displaced PL fragment meeting at least one of the following criteria: intra-articular step or gap >2 mm, extra-articular translation >1.0 cm or angulation >10°; (iii) displaced PL fragments that were relatively simple and an intact bone block (Figure 1A,B,C); (iv) no history of previous injury or surgery in the involved knee joint; (v) a closed fracture with a soft tissue injury less severe than Tscherne type I [14].

**Figure 1:** **Preoperative and intraoperative images.** Preoperative X-ray **(A)** and CT scan **(B, C)** and three-dimensional CT reconstruction **(D)** of a 52-year-old patient, showing the main displaced fragment located at the posterior half of the lateral tibial plateau and a transverse fracture line (case 4). Clinical photographs showing the incision **(E)**, anterior wedge-shaped osteotomy **(F)**, hinging back of the anterior fragment and exposure of the depressed articular segments **(G)** and reduction of the PL fragment with a rasp **(H)**. Reduction was maintained with temporary transcutaneous Kirschner wires, and fluoroscopy was used to verify the reduction **(I, J)**. Before screw placement, the drill bit could be left in the drill hole as a marker for fluoroscopic confirmation of the vector and depth. The most posterior screw was placed first; otherwise, it could not be seen on fluoroscopy **(K, L)**. The position of the plate is shown in **(M, N, O)**.

Based on these criteria, 21 fractures involving the PL corner were screened from 162 surgery patients with lateral tibial fractures from January 2004 to February 2012 in our hospital. Of them, 17 cases treated with open reduction and internal fixation through the anterolateral approach were included in the study (Table 1). However, only 11 cases finally completed the whole experiment. The remaining six patients were excluded from the final analysis: three cases could not be contacted for follow-up (cases 12, 14 and 17), two had a concomitant ligament or meniscal injury that was identified by physical examination under anaesthesia or during the operation (cases 13 and 16) and one was 69 years old with a history of degenerative arthritis (case 15), which would make the results biased. The study design was approved by the institutional review board of the Human Experimental and Ethics Committee in our hospital, and written informed consents were obtained from all patients or their relatives.

**Table 1:** General characteristic of included patients

**Cases**	**Sex**	**Age (years)**	**Cause of injury**	**Comorbidities**	**AL plateau involvement**	**Antibiotic prophylaxis**
1	Male	38	MVA	-	No	No
2	Male	40	MVA	-	No	No
3	Male	23	MVA	-	Yes	Yes
4	Female	52	MVA	-	No	Yes
5	Male	19	Sports	-	No	No
6	Female	53	Fall from height	Diabetes	Yes	Yes
7	Female	22	Sports	-	No	No
8	Male	41	Vehicle accident	-	No	No
9	Female	29	Sports	-	No	No
10	Male	44	MVA	Hypertension	Yes	Yes
11	Male	39	MVA	-	No	No

*AL* anterolateral, *MVA* motor vehicle accident.

### General description and preoperative treatment of included patients

As shown in Table 1, the first 11 cases included consisted of seven males and four females, with age from 19 to 53 years. Of them, seven patients sustained their injuries from motor vehicle accidents (MVAs), three from sports and one from fall from height. Further, case 6 had a diabetes history and case 10 had a hypertension history.

Transcalcaneal traction was done to achieve partial indirect reduction and facilitate healing of the soft tissue preoperatively. The involved legs were kept elevated at least 10 cm higher than the heart and were administered mannitol (20% *m*/*v*, 0.2 g/kg twice a day, intravenous) for 1–3 days to reduce swelling. Surgery was performed when swelling subsided and the skin wrinkled. The mean time from injury to surgery was 3.4 days (range 1–7).

### Surgical procedures

Patients were placed supine on a radiolucent operating table. A tourniquet was used to minimise blood loss and improve fracture visualisation. The knee was flexed to 30°, and a 10–12-cm hockeystick-shaped anterolateral incision was made (Figure 1E). The incision was extended down through the iliotibial band proximally and the fascia of the anterior compartment distally. The tibialis anterior muscle was elevated off the proximal tibia for positioning the plate. A submeniscal arthrotomy was performed to inspect the joint surface, meniscus and cruciate ligament from the anterosuperior aspect.

For the PL pure depression fracture, a cortical window below the area of depression was made. In patients with a PL split and/or depression fracture, we used the indirect reduction method first, but in most situations, anterior wedge-shaped osteotomy was performed and an artificial sagittal cleavage was created, leading to the PL fragment (Figure 1F). To avoid blind osteotomy and to minimise trauma, preoperative computed tomography (CT) images were carefully reviewed. If necessary, a drill bit or guide wire was placed in the tissues as a marker for fluoroscopic guidance before osteotomy. In patients with a sagittal fracture line affecting the AL plateau, the surgical cut was made on the base of the existing anterolateral cleavage in order to reduce further damage. The AL fragment was hinged back on its soft tissue attachment like opening the cover of a book, and the impacted PL articular surface was approached anteriorly (Figure 1G).

The displaced PL fragment was reduced with the help of a bone plunger, rasp or several threaded Kirschner wires (K-wires) (Figure 1H). Depressed articular segments were elevated with a pestle that was inserted as distally as possible, preferably elevating the fragments *en masse* from below. Iliac crest bone grafts or bone graft substitutes were used to maintain the reduction and correct residual depression of the plateau. The AL plateau was then reduced using pointed reduction forceps to re-establish the contour of the anterior cortex and the congruity of the articular surface. Reduction of displaced fragments was maintained with temporary transcutaneous K-wires (Figure 1I,J). The positions of the K-wires were carefully planned to avoid contact with any screws placed in the bone using fluoroscopic guidance (Figure 1I,J).

An anatomically contoured, inverted L-shaped, anterolateral polyaxial locking plate (Numelock II, Stryker, Inc., Mahwah, NJ, USA) was applied because the transverse arm of this plate extends more posteriorly than that of other systems, making it easier to fix the PL fragment (Figures 1O and 2E). We placed screws directly into the PL component, avoiding blind placement. Before screw placement, the drill bit or guide wire could be left in the drill hole as a marker for fluoroscopic confirmation of the vector and depth (Figure 1K,L). The most posterior screw was placed first; otherwise, it could not be seen on fluoroscopy. If the fragment was too lateral to be captured by a screw through the plate, one or two cannulated screws were placed outside the plate to fix the posterior fragment from an anterior direction.

**Figure 2:** **Postoperative images.** Postoperative CT scan **(A, B)**, anteroposterior radiograph **(C)**, lateral radiograph **(D)** and three-dimensional reconstruction **(E)** of a 52-year-old male patient, showing satisfactory restoration of congruity of the articular surface and alignment of the lower extremity (TPA 88°, PSA 5.7°, articular step-off <2 mm). Note that the PL fragment was fixed with the anterolateral polyaxial locking plate.

The plate was inserted by sliding it underneath the muscle to minimise disruption of blood supply. Metaphyseal locking screws were placed subchondrally to buttress the elevated articular surface, and diaphyseal screws were placed via stab incisions. The position of the plate is shown in Figure 1M,N,O.

### Postoperative management

The postoperative patients underwent continuous passive movement exercises under the supervision of a physical therapist. No weight bearing was allowed for a minimum of 4 weeks. Toe-touch weight bearing was started at 4–8 weeks, with subsequent progression depending on the radiographic findings.

The clinical and radiographic outcomes were recorded (Figure 2). Clinical evaluation parameters included operation time, incision length (IL; not counting the stab incisions for distal screw placement), range of motion (ROM), Hospital for Special Surgery (HSS) knee score [15], time of union and complications. The HSS is an extensive, internationally acknowledged assessment instrument, developed for follow-up evaluations of knee arthroplasty, including pain and function components. Radiographic evaluation included the tibial plateau angle (TPA) representing the coronal alignment of the proximal tibia, the lateral posterior slope angle (PSA) reflecting the sagittal alignment of the proximal tibia and articular step-off reduction. Reduction was considered to be satisfactory with articular step-off <2 mm, TPA 87° ± 5° and PSA 9° ± 5°. Imaging examination was performed once immediately after surgery and then once a month until the fracture healed. Radiographic outcomes, HSS and ROM were measured at the final follow-up (Figure 3).

**Figure 3:** **Radiographic outcomes, HSS and ROM.** Lateral radiograph **(A)** at 9 months postoperatively with the knee flexed to 85°, showing complete fracture healing with a satisfactory range of motion. The flexion and extension functions of the knee performed no abnormality in the last follow-up **(B, C)**.

## Results

### Immediate characteristics after surgery

According to the data in Table 2, 72.7% patients (8/11) accepted the anterior osteotomy for visualisation. The means of TPA, PSA and articular step-off were 85.5°, 8.1° and 1.2 mm, respectively. The mean operation time was 82 min (range 62–105 min), the mean incision length was 11 cm (range 10–14 cm) and the mean time from injury to surgery was 3.4 days.

**Table 2:** Immediate postoperative patient characteristics

**Cases**	**Anterior osteotomy for visualisation**	**Reduction**			**OT (min)**	**IL (cm)**	**AO/OTA classification**	**Time from injury to surgery (days)**
		**TPA (deg)**	**PSA (deg)**	**SF (mm)**				
1	Yes	85	7.3	1	62	11	41-B2.2(3)	3
2	Yes	84	7.1	0	75	10	41-B2.2(4)	4
3	No	82	8.4	2	100	14	41-B3	4
4	No	88	5.7	0	105	14	41-B3.1(2)	3
5	Yes	85	6	1	70	12	41-B2.2(4)	1
6	Yes	91	9.2	0	75	10	41-B3	2
7	Yes	81	11.4	0	95	14	41-B1.1(4)	7
8	Yes	87	12	2	70	10	41-B1.1(4)	2
9	Yes	81	8.2	1	80	10	41-B2.2(4)	3
10	No	85	6.1	5	105	13	41-B3	3
11	Yes	91	8	1	65	10	41-B2.2(4)	5
Mean	-	85.5	8.1	1.2	82	11.6	-	3.4

*TPA* tibial plateau angle, *PSA* posterior slope angle, *SF* articular step-off, *OT* operation time, *IL* incision length.

### Clinical outcomes at final follow-up

Based on Table 3, the mean follow-up period was 27.1 months (range 18–44 months). The mean HSS score was 91.2 (range 86–96), ROM was 97° (range 75°–125°) and the fracture union was observed at a mean postoperative time of 3.7 months (range 3–6 months). The means of TPA, PSA and articular step-off were 87.2°, 8.3° and 1.2 mm, respectively. The reduction was satisfactory in 10 patients, except for one patient who had a radiographic articular step-off of 5 mm (case 10).

**Table 3:** Clinical outcomes at final follow-up

**Case**	**FU (months)**	**SS**	**ROM (E-F)**	**HSS score**	**UT (months)**	**Reduction**		
						**TPA (deg)**	**PSA (deg)**	**SF (mm)**
1	25	Excellent	0–95	95	3	84	7.0	1
2	18	Good	0–125	94	4	87	7.1	0
3	36	Good	5–80	88	3	83	8.4	2
4	20	Excellent	0–120	88	3	88	5.7	0
5	20	Excellent	0–100	93	4	83	6.6	1
6	18	Good	5–100	90	5	92	9.3	0
7	35	Good	5–105	90	6	80	11.4	0
8	22	Fair	0–85	86	3	103	13	2
9	24	Excellent	0–100	92	3	86	8.2	1
10	40	Good	0–85	91	4	86	6.2	5
11	40	Good	0–75	96	3	87	8.1	1
Mean	27.1	-	97.3	91.2	3.7	87.2	8.3	1.2

*FU* follow-up, *SS* subjective satisfaction, *ROM* range of motion, *E-F* extension to flexion, *HSS* Hospital for Special Surgery, *UT* union time, *TPA* tibial plateau angle, *PSA* posterior slope angle, *SF* articular step-off.

### Complications after surgery

Of the 11 patients, three patients developed complications after surgery: one got superficial infection, one hardware irritation and one secondary valgus deformity. The patient with a superficial infection was treated successfully with antibiotics and debridement (case 5). The second patient underwent hardware removal surgery after 1.5 years with no further complications (case 9). The last patient with secondary valgus deformity with TPA of 103° expressed subjective satisfaction with the outcome (case 8). Therefore, the AL approach was successfully conducted in the fracture treatment.

## Discussion

A PL tibial plateau fracture is uncommon and is regarded as a split fracture and/or compression in the posterolateral aspect of the tibial plateau [3,16]. The AO/OTA classification system [2] classifies posterolateral tibial plateau fractures as being partial articular (41-B). Adding a number in parentheses depicts the posterior articular surface in a more comprehensive way: 41-B1.1(4) illustrates a partial articular split fracture of the proximal tibial lateral surface on the posterior aspect on the frontal plane, 41-B2.2(4) illustrates a proximal tibial partial articular depression fracture of the lateral plateau on the posterior aspect, 41-B3.1(2) illustrates a proximal tibial partial articular split-depression fracture of the lateral plateau on the posterolateral part; the patients suffering from tibial fractures involving the anterolateral plateau, without obvious displacement, in our study were also included in the AO/OTA classification of posterolateral tibial plateau fractures because of the similar therapy, and the fractures were named as lateral plateau fractures with PL corner involvement based on the displacement characteristics. We focus on these types of fractures because they have similar displaced PL fragments which are usually fixed using the posterior approach, but the best option is still controversial and unclear.

As for the treatment, many doctors argued that these fractures should be conducted through the PL approach because of the easy exposure of the surgical area or convenient fixation of the fractures [17,18]. Exactly, the PL approach is undoubtedly the best choice for cases which must be treated from the posterolateral aspect [4]. For example, most PL platform fractures with shift, especially fractures with severe crush and inversion shift, can usually be treated with the PL approach; the AL approach cannot fully expose the surgical area and accurately restore and stably fix the fractures. As for other types of fractures which can be treated by either the AL approach or the PL approach, the AL approach can generally avoid surgery damages on important nerves and vessels and also lead to less complications in comparison with the PL approach because the PL approach is usually a traumatic procedure, which may damage the related nerves and vessels nearby anatomically [6,19]. Further, isolated posterior approaches do not allow sufficient visual control of fracture reduction, especially for complex fractures. However, anatomically, the AL approach can generally avoid surgery damages on important nerves and vessels.

Based on the disadvantages of the PL approach and the obvious advantages of the AL approach, we retrospectively studied 11 patients with a PL plateau fracture. The obvious features of these cases were all classified into a relatively simple and intact PL fragment. The characteristics permitted the anterolateral polyaxial locking plate to be tightly fixed to the fracture block with at least one or two locking screws. Then, with the help of the lag screws from the anterior buttress plate, fixation could supply necessary stability for the early mobilisation of the posterolateral fracture plate. In our treatment of PL tibial plateau fractures with the AL approach, there were slight complications such as a superficial infection, hardware irritation and secondary valgus deformity. However, no severe perioperative complications occurred, for instance, deep venous thrombosis and pulmonary embolism. Our results keep in line with previous reports that the anterior approach can be used to treat PL tibial plateau fractures with good clinical outcomes [3].

The result of our study is encouraging, but there are still some contraindications to the application of the AL approach for the treatment of PL plateau fractures. In comminuted PL plateau fractures with multiple and tiny displaced fragments, it is difficult to obtain and maintain anatomical reduction with the use of the AL approach. In this case, even with careful preoperative planning and the use of intraoperative fluoroscopy, it is not always possible to fix all fragments and avoid contact between the screws and K-wires [4]. In addition, if the fracture plate cannot be fixed by the locking screws from the polyaxial locking plate system, the support function of the lag screws from the anterior buttress plate cannot also supply enough stability. Besides, the AL approach is not adaptable to cases with neurovascular injury or soft tissue interposed in the fracture fragments, and these types of injury need broad exposure using the posterior approach and complex repair surgery or removal of interposed tissues.

Finally, the AL approach for the treatment of PL plateau fractures is only suitable for the PL fracture plate which is relatively simple and intact, without inverted displacement. The key technical essential affecting the success of the whole surgery is fixation using the polyaxial locking plate and screws which can catch the PL fracture fragment. If the locking screws from the polyaxial locking plate system cannot tightly lock the fracture plate, the lag screws alone are not enough for stability. Therefore, cast protection after surgery will be necessary for such conditions. Moreover, knee hyperextension indirect reduction and bone window reduction techniques should be used in combination [3], if necessary, and anterolateral wedge osteotomy can be used for the reduction of PL fracture fragments visually. It is certain that the AL approach for the treatment of PL plateau fractures is safe and effective if the indications and internal fixation method are properly and carefully screened as above.

## Conclusions

The AL approach is safe and effective for the treatment of patients with lateral tibial plateau fractures involving the PL corner, especially for fractures merged with relatively simple and intact PL corner displacement (depression and/or split). The key factor in surgery is rigid fixation to the PL fracture fragment using the polyaxial locking plate system.

## Competing interests

The authors declare that they have no competing interests.

## Authors’ contributions

DM participated in the design of this study. TY carried out the study, together with AC, collected the important background information and drafted the manuscript. DM conceived of this study, participated in the design and helped draft the manuscript. All authors read and approved the final manuscript.
